The article "The Effect of Deep Learning-Based QSM Magnetic Resonance Imaging on the Subthalamic Nucleus" was retracted in 2023. Reasons: signs of a paper mill; suspected computer-generated content; unreliable results or conclusions; concerns about the data.

# The Effect of Deep Learning-Based QSM Magnetic Resonance Imaging on the Subthalamic Nucleus

**DOI:** 10.1155/2021/8554182

**Published:** 2021-09-15

**Authors:** Yuanqin Liu, Qinglu Zhang, Lingchong Liu, Cuiling Li, Rongwei Zhang, Guangcun Liu

**Affiliations:** ^1^Department of Neurosurgery, Shandong Provincial Qianfoshan Hospital, Cheeloo College of Medicine, Shandong University, Jinan, Shandong 250014, China; ^2^Department of Special Examination, Shandong Provincial Third Hospital, Cheeloo College of Medicine, Shandong University, Jinan, Shandong 250031, China; ^3^Department of Medical Imaging Shandong Provincial Qianfoshan Hospital, Cheeloo College of Medicine, Shandong University, Jinan, Shandong 250014, China

## Abstract

In order to study the influence of quantitative magnetic susceptibility mapping (QSM) on them. A 2.5D Attention U-Net Network based on multiple input and multiple output, a method for segmenting RN, SN, and STN regions in high-resolution QSM images is proposed, and deep learning realizes accurate segmentation of deep nuclei in brain QSM images. Experimental results show data first cuts each layer of 0 100 case data, based on the image center, from 384 × 288 to the size of 128 × 128. Image combination: each layer of the image in the layer direction combines with two adjacent images into a 2.5D image, i.e., (*It* − *m It*; *It* + *i*), where *It* represents the layer *i* image. At this time, the size of the image changes from 128 × 128 to 128 × 128 × 3, in which 3 represents three consecutive layers of images. The SNR of SWP I to STN is twice that of SWI. The small deep gray matter nuclei (RN, SN, and STN) in QSM images of the brain and the pancreas with irregular shape and large individual differences in abdominal CT images can be automatically segmented.

## 1. Introduction

Medical image segmentation is the key to use the medical image for computer-aided diagnosis. In recent years, deep learning has achieved remarkable results in the field of computer vision, and convolutional neural network (CNN) has also achieved significant breakthroughs in image segmentation [1]. Iron deposits in red nucleus (RN), substantia nigra (SN), and subthalamic nucleus (STN) are considered to be responsible for the development of Parkinson's disease, accurate division of these cores is the premise of a quantitative study of iron deposition in cores, which is of great significance [2]. However, accurate segmentation of the nuclear mass is difficult due to its small volume and poor contrast with surrounding tissues. The thalamus is the brain's relay station, receiving all sensory signals except for smell and sending them to the cerebral cortical region. The thalamus can be divided into multiple nuclei, and each nucleus has a specific function [3]. There are connections between the nuclei and specific cortical regions or they act as relays between cortical connections. Many neurological diseases are closely related to the damage of the thalamic nucleus, such as Alzheimer's disease, Parkinson's disease, schizophrenia, epilepsy, and carbuncle. Deep brain stimulation surgery can effectively treat these diseases by implanting pacemakers into specific nuclei of the thalamus [4]. Therefore, accurate thalamic segmentation is of great value and significance for brain cognition research, mechanism research, diagnosis and treatment of neurological diseases, and other fields. Quantitative magnetic resonance mapping (QSM) has many advantages, such as high resolution, good contrast, and no radiation, and is widely used in brain cognition research and diagnosis and treatment of neurological diseases [5]. Magnetic resonance imaging provides a good basis for the accurate segmentation of the thalamus. Manually segmenting MRI images is a time-consuming and cumbersome task. Automatic and accurate thalamic segmentation is of great value for subsequent diagnosis and treatment [6]. Magnetic-sensitive correlation sequences also have some drawbacks, including signal loss, distortion, and local field strength inconsistency. In particular, at high field strengths, nonlocal magnetic sensitization effects (causing halo artifacts) may lead to the edge blur of the STN. Since the STN slopes in 3 planes and has a small structure, these halo artifacts need to be quantified and corrected before pinpointing the STN.

She et al. proposed that the human brain has numerous neurons composed of cell bodies and axons. The human brain tissue can be divided into three types: the gray matter composed of cell bodies, the white matter composed mainly of axons, and the cerebrospinal fluid (CSF) between the gray matter and white matter. The reflection intensity of RF magnetic field energy varies with the water content of different tissues, so MRI images are reflected in different image intensities [7]. Li et al. proposed that some gray matter structures in the brain, such as the caudate nucleus, globus pallidus, and thalamus, are closely related to brain diseases such as Parkinson's disease, carbuncle epilepsy, and Alzheimer's disease. The main clinical treatment of these diseases is the use of drugs and stereotactic neurosurgery. With the development and combined application of stereotactic technology, computer technology, and imaging technology, stereotactic surgery has gradually become the main means for the treatment of such neurological diseases [8]. Lancelot et al. proposed that the common target area in clinical DBS surgery is located in the deep nucleus of the brain, among which a key common site is the thalamus. The thalamus is the brain's relay station, receiving all sensory signals except for smell and sending them to the cerebral cortical region. The thalamus can be divided into multiple nuclei, and each nucleus has a specific function. Nuclear clusters produces connections with specific cortical regions or act as relays between cortical connections [9].

The Rn, SN, and STN regions in high-resolution QSM images are segmented by 2SD Attention U-Net based on multi-input and multioutput. In addition, transfer learning of low-resolution data is used to solve the problem of the low number of high-resolution QSM images. We studied the conditions of transfer learning, and the results proved data first cuts each layer of 0 100 case data, based on the image center, from 384 × 288 to the size of 128 × 128. Image combination: each layer of the image in the layer direction combines with two adjacent images into a 2.5D image, that is, (*It* − *m It*; *It* + *i*), where *It* represents the layer *i* image. At this time, the size of the image changes from 128 × 128 to 128 × 128 × 3, in which 3 represents three consecutive layers of images. When all model parameters were iteratively fine-tuned, the transfer model could achieve the best segmentation effect in a relatively short period of time, and the effect was close to that of artificial segmentation [10].

## 2. Deep Learning-Based Thalamus Segmentation Method

Characterized by strong soft-tissue contrast, high spatial resolution, and the absence of known health risks, magnetic resonance imaging is often the method of choice for structural brain analysis. Quantitative brain MRI has been widely used to characterize brain diseases such as Alzheimer's disease, epilepsy, schizophrenia, and multiple sclerosis. MRI signal contains phase information and amplitude information. Traditional MR imaging methods mostly use amplitude information while ignoring phase information [11, 12]. By preprocessing the phase information obtained, we can obtain the information reflecting the local magnetic field variation caused by the difference in the magnetic susceptibility between tissues. Quantitative susceptibility imaging technology uses the phase information of the signal to obtain the information of the local magnetic field of the tissue and then through the physical relationship between the magnetic field and the susceptibility to reverse the distribution of the magnetic susceptibility image. Usually, magnetic resonance data is obtained by Gradient echo GRE. In the reconstruction process of quantitative magnetic susceptibility image, the data is firstly preprocessed (magnetic field image fitting and phase unwinding), then the background field is removed, and finally the magnetic susceptibility inversion is carried out. The magnetic distance of GRE is *T*2^*∗*^ sensitive to iron, and the phase is proportional to the magnetic field generated by iron in the tissue. The magnetic distance and phase signal of the same part are affected by the distribution of iron in the surrounding tissue due to the high iron content in Sn, Stn, and Rn regions [13, 14].

The region-based thalamic segmentation method includes the region growing method, the active contour model method, and the K-mean method.

1. Zone growing is a method of gradually growing groups of pixels or areas into larger areas. Firstly, an initial point in the region to be segmented is found as the growth seed. By making appropriate growth and similarity rules, properties similar to the seed in the neighboring region, such as gray level, intensity, and texture color, are combined into the region where the seed is located. These new elements are used as a new seed set and the above process is repeated continuously until the conditions for stopping growth are met or the pixels that do not meet the conditions are met [15, 16].
2. Methods based on the active contour model are mainly divided into two categories: Parametric active contour model (Snake model) and geometric active contour model (level set method). The snake model is originally based on the minimum energy curve to find the boundaries of different regions. The method is mainly used to segment a single structure, such as the ventricle or the hippocampus. The snake model requires that the initial contour be similar to the target contour. Level set method: later, researchers used the level set method to segment brain MRI images.
3. K-mean and method: Firstly, K clustering centers are randomly selected to calculate the distance between other pixels in the image and the clustering center, divide the pixels into the clustering center closest to it, and then point to all the pixels in each cluster. The average value of all the pixels in each cluster is used as the new clustering center. Calculate and recluster the distance from all the pixels to the new cluster center. It then iteratively continues until the pixels in each cluster are essentially unchanged, and finally, the segmented image is obtained. This method mainly uses the difference of image gray value to distinguish categories, so it is susceptible to the influence of image texture factors, with low computational efficiency, and the pixels in the image can only belong to one category [17, 18].

### 2.1. Medical Image Segmentation Method Based on Convolutional Neural Network

Deep learning (DL) is a new machine learning algorithm that simulates human thinking. In 1998, LeCun et al. proposed a Convolutional neural network (CNN) and applied the backpropagation algorithm to the learning process of a feedforward multilayer neural network to recognize handwritten numbers. But with the deepening of the network layer number, the problem of gradient disappearance will appear in the multilayer network. Until 2006, Hinton's team solved the problem of gradient disappearance of backpropagation algorithm, which made a breakthrough in deep learning in image target recognition, classification, and prediction. In recent years, with the development of deep learning, researchers are increasingly using natural image semantic segmentation models to solve the segmentation tasks of medical images. When the convolutional neural network is used to automatically segment medical images, the network model is firstly trained with the data in the training set, and the parameters in the model are obtained. At the same time, the data in the validation set are used to select the optimal segmentation model. Finally, the data in the test set was input into the optimal model for segmentation, and the output probability graph was binarized to obtain the final target region. The process is shown in Figure 1.

As can be seen from Figure 1, the quality of the model is the key factor that determines the segmentation result. The quality of the model depends largely on the structure of the model and the type of loss function used in the training process. Several typical medical image segmentation models and loss functions will be introduced in the following sections.

The most commonly used loss function in image segmentation is the perpixel crossover function as follows:

(1) $$\begin{array}{c} CL\left(\theta \right)=\sum_{i=1}^{N}G_{i}\;\log\;P\left(X_{i};\theta \right)+\left(1-G_{i}\right)\log\;P\left(X_{i};\theta \right), \end{array}$$

where *CL*(*θ*) represents the energy value, the data representing the gold standard graph *P*(*X*_*i*_; *θ*) represents the prediction probability graph data. As can be seen from equation (1), the loss function of cross linearly separately evaluates the class prediction of each pixel vector and then averages all pixels, so the pixels in the image are equally learned [19, 20]. However, the imbalance of categories often occurs in medical images. As a result, the training will be dominated by classes with more pixels, and it is difficult to learn the features of smaller objects, which reduces the effectiveness of the network. In order to reduce the contribution of the weight of the well-segmented sample and make CNN focus more on the hard-to-segment sample, a term (1 − *P*(*X*_*i*_; *θ*))^*γ*^ is added to the cross-child loss as follows:

(2) $$\begin{array}{c} FL\left(\theta \right)=\sum_{i=1}^{N}a{\left(1-P\left(X_{i};\theta \right)\right)}^{\gamma }G_{i}\;\log\;P\left(X_{i};\theta \right), \end{array}$$

where *FL*(*θ*) represents the energy value, “represents the data of the gold standard graph, and *P*(*X*_*i*_; *θ*) represents the prediction probability.

Dice Loss can measure the overlap of divided areas. This indicator ranges from 0 to 1, where “1” indicates complete overlap. Its calculation is shown in the following equation:

(3) $$\begin{array}{c} DL=\frac{2\times G_{i}\cap P\left(X_{i};\theta \right)}{p\left(X_{i};\theta \right)+G_{i}}. \end{array}$$

Jaccard Loss is a statistic used to compare the similarity and diversity of predicted images and gold standard images. It is defined as the size of the intersection region divided by the size of the union region as follows:

(4) $$\begin{array}{c} JL=\frac{G_{i}\cap P\left(X_{i};\theta \right)}{G_{i}\cup P\left(X_{i};\theta \right)}. \end{array}$$

There are many evaluation indexes used in medical image segmentation. In this paper, DSC (Dice similarity coefficients, precision, recall) and DSC (Dice similarity coefficients, precision, recall) are introduced.

Similarity coefficient (DSC) is used to measure the similarity between the binary graph *P* predicted by segmentation network and the gold standard *G* as follows:

(5) $$\begin{array}{c} \text{DSC}=\frac{2\times S\left(P\cap G\right)}{S\left(P\right)+S\left(G\right)}. \end{array}$$

Accuracy rate, also known as the precision ratio, is used to calculate the proportion of true positive samples among all predicted positive samples as follows:

(6) $$\begin{array}{c} \text{precision}=\frac{\text{TP}}{\text{TP}+\text{FP}}. \end{array}$$

The positive samples predicted to be positive by the TP (true positive) model, in this experiment, represent all the regions in *P* with pixel value of 1, and the number of pixels in *G* with pixel value of 1; FP (the negative sample predicted by the false positive model), in this experiment, represents the number of pixels in all the regions with pixel value 1 in *P* and the number of pixels with pixel value 0 in *G*. The recall rate is also called recall rate, and the percentage of positive samples predicted by the model is calculated as follows:

(7) $$\begin{array}{c} \text{recall}=\frac{\text{TP}}{\text{TP}+\text{FN}}, \end{array}$$

where the positive samples predicted by FN (false negative) model are negative, which in this experiment represents the number of pixels in all the regions with pixel values of 0 (P) and 1 (P) in all regions.

### 2.2. Based on Image Postprocessing Technology

QSM is an image postprocessing technique that can be used on GRE phase images of the SWI sequence to solve the halo artifact problem. The linear correlation between QSM imaging and brain tissue iron concentration has more ladder gradients than SWI and more accurate estimation of tissue iron concentration, thus allowing better identification of iron-rich structural boundaries with the surrounding structure 35. The application of QSM in STN localization may have good prospects.

## 3. Experimental Analysis

Due to the high cost of QSM image acquisition, the amount of high-resolution data in the experimental data is limited and there are many low-resolution data. In this chapter, the method of transfer learning is used to make the low-resolution data provide part of the features so that the model can be more rapid and accurate in the segmentation of the core groups in high-resolution data. This study has been approved by the local ethics committee, and all participants have signed the informed consent. The low-resolution data used in this study were head MRI images of 100 subjects (43.67 and 15.65 years old, 45 males, and 55 females). All participants were scanned using a Siemens Clinical 3T Magnetic resonance imaging (MAGNETOM Trio TIM, Siemens Healthcare, Erlangen, Germany) equipped with a 12-channel head coil. QSM is collected by 3D multi-echo GRE sequence, and the specific scanning parameters are shown in Table 1.

Before the image is input into the network, the low-resolution data are preprocessed in the experiment; the process is as follows:

1. Data splitting: Data of 100 cases were randomly divided into training set (70 cases), verification set (10 cases), and test set (20 cases).
2. Data screening and one-hot coding: In fact, there are very little data containing ROI in each data case. In order to reduce interference information, data of training set and verification set need to be screened. All the layers containing ROI and some layers without ROI were selected along the direction of the layer (in the layer without ROI, 3 layers were randomly selected from each of the 5 layers near both ends of the region containing ROI, a total of 6 layers), as the subsequent training data input into the network. Then, the label of all data is one-hot coded.
3. For the first time, each layer of 0 100 cases of data is clipped from 384 × 288 to 128 × 128 based on the center of the image.
4. Image combination: The image of each layer along the direction of the layer is combined with two adjacent images to form a 2.5D image, namely, (*IT* − *m IT*; *It* + *I*), where *It* represents the *i*-layer image. At this time, the size of the image changed from 128 × 128 to 128 × 128 × 3, where 3 represents the image of three successive layers.
5. Data amplification: During the training process, with each iteration, data amplification was carried out on the samples of the extracted training set and verification set. The amplification methods included random translation within the range of 10 pixels, random stretching within the range of 10%, and random rotation within 5 degrees.
6. The second data cutting: After data amplification, the image will contain some information that does not belong to the image, as shown in Figure 2. Therefore, we will cut the data for the second time, also taking the image center as the base point, cutting it from 128 × 128 to 96 × 96. In magnetically sensitive sequences, SWI has good CNR; SWPI has a signal-to-noise ratio greater than T2 ∗ STN for STN SNR, 2 times SWI and 3.5 times T2∗WI, second only to QSM. The CNR of QSM is superior to T2, FSE-T2WI, T2∗WI, SWPI, and SWI, to clearly show the portions of STN above and below SN and reduces halo artifacts generated by the GRE sequence. Therefore, magnetic-sensitive sequences and image reconstruction sequences may replace T2WI.

Firstly, a segmentation Model L (Model L) was trained to segment RN, SN in low-resolution brain images. Then, the Model's parameters were transferred to the segmentation network of high-resolution brain MRI images as initial parameters, so as to achieve the goal of segmenting RN, SN, and STN with fewer high-resolution brain QSM images. When using low-resolution QSM images to train 2SD multi-input in-depth supervision Attention U-Net, it is necessary to continuously optimize the network parameter *θ*. In each iteration, 20 preprocessed samples are randomly selected from the training samples and input into the network after data amplification. The energy value is calculated by the energy function between the output results and the gold standard; then, the energy value is input to the optimizer to optimize so that the network updates the weight *W* and deviation B through the backpropagation algorithm. The basic energy function used in the experiment is Tversky loss, as shown in equation (8), and *β*=0.7 is set in this experiment:

(8) $$\begin{array}{c} TL\left(\theta \right)=\overset{n}{\underset{i=1}{\sum }}\frac{G_{i}\cap P\left(X_{i};\theta \right)}{G_{i}\cap P\left(X_{i};\theta \right)+a|G_{i}-P\left(X_{i};\theta \right)+\beta |P\left(X_{i};\theta \right)-G_{i}|}, \end{array}$$

where *TL*(*θ*) represents the energy value, “represents the data of the gold standard graph *P*(*X*_*i*_; *θ*) represents the data of the prediction probability graph. *a*=*β*=0.5 can be properly set by observation. In this case, Tversky loss is Dice loss. When *a*=*β*=1 is set, Tversky Loss is Jaccard Loss. *A* and *β* controlled for false negatives and false positives, respectively. By adjusting the values of *a* and *β*, we can control the tradeoff between false positives and false negatives. According to these segmentation results, the energy function was calculated respectively with the gold standard, and different weights were allocated for summation. In the training process, the energy function was jointly optimized. The calculation method of the total loss function *Loss* is shown as follows:

(9) $$\begin{array}{c} \text{Loss}=a\times {\text{loss}}_{1}+b\times {\text{loss}}_{2}+c\times {\text{loss}}_{3}+d\times {\text{loss}}_{4}. \end{array}$$

Loss_*n*_ (*n* = 1, 2, 3, 4) are the energy functions obtained from the gold standard of the four outputs from top to bottom and their corresponding sizes. *a*, *b*, *c*, and *d* represent the weights of the four energy functions, respectively; through experiments, *a* = 0.6, *b* = 0.2, *c* = 0.1, and *d* = 0.1 were set in this paper.

In order to quantitatively evaluate the segmentation effect of the Model network on Rn and SN regions, the results of the network output and the segmentation results of the gold standard were used to calculate DSC in the experiment. The segmentation results of each case of data in the test set and the DSC statistics of the gold standard were represented by a discount graph, as shown in Figure 3.

As can be seen from Figure 3, the median of the RN region segmented by the model and the gold standard DSC is about 0.83, but it contains three smaller singular values, so the final mean value is only 0.78. The median of the SN region segmented by the model and the gold standard DSC is about 0.76, which contains a small singular value, so the final mean value is only 0.74. In general, although the segmentation results of the model for Rn and Sn are different from those of the gold standard, the core group can be roughly segmenting.

In this study, we segmented the deep gray matter nuclei in low-resolution QSM images and high-resolution QSM images using the multi-input and multioutput Attention U-Net network and achieved relatively accurate segmentation effects. As MRI develops, it is gradually applied to STN positioning, including direct positioning of wearing framework and fusion positioning with CT images. In order to individualize and accurately implant the electrodes into the sensory movement part (dorsolateral region) of STN, it is required to make a clear division of the nuclear group boundary on the MRI image and ensure the minimum geometric distortion of the image, but the current effect is not ideal

## 4. Conclusions

With the widespread use of deep brain stimulation surgery, accurate positioning of the thalamus has become a key link to improve the accuracy of electrode placement. Preoperative imaging is indispensable as a core means to identify the target thalamus. By introducing dense connection in DenseNet, residual learning in ResNet, and bottleneck design in InceptionNet, combining with practical application scenarios of thalamic MRL image segmentation, magnetic-sensitive correlation sequences also have some drawbacks, including signal loss, distortion, and local field strength inconsistency. In particular, at high field strengths, nonlocal magnetic sensitization effects (causing halo artifacts) may lead to the edge blur of the STN. Since the STN slopes in 3 planes and has a small structure, these halo artifacts need to be quantified and corrected before pinpointing the STN. For the first time, cut each layer of 0–100 cases of data, and take the image center as the base point to change the image from 384 × 288 cut to 128 ×128. Image combination: combine each layer image along the layer direction with two adjacent images to form a 2.5D image, i.e., (It–m It; It+i), where it represents the image of layer I. At this time, the size of the image is changed from 128 × 128 to 128 × 128 × 3, where 3 represents 3 consecutive layers of images. The RDU-NET network model is proposed, which has certain practical value and has reference significance for related research. The experiment proves that when the transfer learning is used to train the transfer model, the training time is greatly reduced, and when all the transfer parameters are fine-tuned in the iterative process, the model has the best segmentation effect on the core group and achieves the segmentation effect close to that of the artificial one. The algorithms are all based on 2SD images for research, which loses more spatial information. Therefore, 3D network will be directly used to solve the problem of medical image segmentation in future research. In addition, it can be combined with the detection network in the future experiment, and the approximate target region can be detected first and then segmented.

## Figures and Tables

**Figure 1:** The flowchart of training and testing methods for the convolutional neural network (CNN) segmentation model in medical images.

**Figure 2:** Flowchart of image preprocessing.

**Figure 3:** DSC boxplot of Rn and SN segmentation results.

**Table 1:** Experimental parameters.

Gender differences	Age	Recovery time (ms)	First wave of time (ms)	Wave echo interval time (ms)	Frequency
Man	43.67 ± 15.65	60	6.8	6.9	8
Women	40.23 ± 13.62	46	5.6	4.8	6

## Data Availability

The data used to support the findings of this study are available from the corresponding author upon request.
